# Harman and norharman, metabolites of the entomopathogenic fungus *Conidiobolus coronatus* (Entomophthorales), affect the serotonin levels and phagocytic activity of hemocytes, insect immunocompetent cells, in *Galleria mellonella* (Lepidoptera)

**DOI:** 10.1186/s13578-019-0291-1

**Published:** 2019-03-25

**Authors:** Anna Katarzyna Wrońska, Mieczysława Irena Boguś

**Affiliations:** 1 Witold Stefański Institute of Parasitology, Polish Academy of Sciences, Twarda 51/55, 00-818 Warsaw, Poland; 2 BIOMIBO, Ul. Strzygłowska 15, 04-872 Warsaw, Poland

**Keywords:** Serotonin, Phagocytosis, Harman, Norharman, Insect hemocytes

## Abstract

**Background:**

Although the β-carboline alkaloids harman and norharman are considered as plant metabolites, they can also be secreted by fungi such as the entomopathogen *Conidiobolus coronatus*. Norharman and harman are also known to be reversible competitive monamine oxidase inhibitors, which increase serotonin concentrations in tissues. In addition, these alkaloids are able to bind to serotonin receptors, an important immune regulatory molecule in both vertebrates and invertebrates. In insects, serotonin modulates hemocyte phagocytosis, nodule formation and the populations of hemocyte classes. The present study examines whether harman and norharman may influence the phagocytic activity of insect hemocytes by regulating serotonin levels.

**Results:**

Significantly greater serotonin levels and hemocyte phagocytic activity were observed after 24 h of exposure to food contaminated with harman and norharman. Similar responses were noticed 1 h after topical application or addition to in vitro hemocyte cultures. Observations and measurements performed 24 h later revealed decreased responses, suggesting decomposition and/or exertion of alkaloids and/or serotonin. Harman and norharman influenced the activity of *Galleria mellonella* plasmatocytes and the granulocyte cytoskeleton. Disturbances in hemocyte network formation, abnormal cell shape, naked nuclei, cell aggregates, fragments of disintegrated cells, interrupted cell membrane continuity and actin condensation in cells were observed.

**Conclusion:**

Our findings may have a considerable impact on research concerning insect physiology, parasitology, immunology and biocontrol of pests. They confirm for the first time that harman and norharman (metabolites of the entomopathogenic fungus *C. coronatus*) elevate serotonin levels in *G. mellonella* hemocytes, thus potentially stimulating their phagocytic activity. Our studies shed light on the mechanisms underlying the interaction between innate insect immune responses and entomopathogen metabolites.

**Electronic supplementary material:**

The online version of this article (10.1186/s13578-019-0291-1) contains supplementary material, which is available to authorized users.

## Background

The β-carboline alkaloids were originally isolated from *Peganum harmala* (Zygophillaceae, Syrian Rue), a traditional herbal drug commonly used as an emmenagogue and abortifacient in the Middle East and North Africa [1]. During the last two decades, the major bioactive constituents of the drugs have been isolated from various terrestrial plants, these being numerous simple and complicated β-carboline alkaloids with saturated or unsaturated tricyclic ring systems. Of these agents, the most widely described are norharman and harman [2], with a wealth of data regarding their impact on mammals being recorded in the literature. Norharman and harman are known to be reversible competitive monamine oxidase (MAO) inhibitors: norharman preferentially inhibits MAO-B, whereas harman inhibits MAO-A [3]. In addition to their interaction with enzyme systems, various receptor proteins are also important targets for β-carboline. Since the first reports that β-carboline alkaloids are able to bind to serotonin (5-HT) receptors of isolated tissue [4], this relationship has been the subject of many investigations. One study found that both harman and norharman bind to 5-HT receptors, causing an increase of 5-hydroxyindoleacetic acid (5-HIAA) and homovanillic acid (HVA) levels in rat brain [5]. It is important to understand the effect of these compounds on insects.

There is a growing need to reduce the amounts of chemical insecticides, and in response to this, entomopathogenic fungi are becoming increasingly popular as bio-insecticides, as the use of naturally or artificially-introduced organisms to reduce arthropod populations can ensure greater safety for consumers, plants and the environment. This is especially important for organic farming, where there is need to extend the range of alternatives available for controlling harmful insects [6]. Although the use of insecticidal fungi in crop and forest protection has so far been limited, more than 100 species of fungi are currently under review as candidates for reducing the numbers of arthropod pests [7].

The process of infection by an entomopathogenic fungus begins with its adhesion to an insect body; this is followed by the secretion of enzymes that hydrolyze the epidermis of the insect. The most important enzymes secreted by entomopathogenic fungi in this regard are lipases, proteases and chitinases, which are produced sequentially, reflecting the order of the substrates they encounter [8]. The consequent tissue destruction, exhaustion of nutrients or the effect of fungal toxins results in the death of the host. A number of toxic compounds such as small secondary metabolites, cyclic peptides and macromolecular proteins have been isolated from the filtrate of entomopathogenic fungi [9]. Some species of entomopathogenic fungi are capable of producing alkaloids.

The first evidence that the entomopathogenic fungus *C. coronatus* produces two toxic β-carboline alkaloids, harman and norharman, was given by Wrońska et al. [10]. In this study, the highest amounts of norharman and harman were found in cell-free filtrates of MM (minimal medium) post-incubation medium, and that both alkaloids delayed *Galleria mellonella* pupation and adult eclosion. In addition, harman and norharman were found to increase serotonin concentration and decrease MAO-A level in the heads of wax moth larvae, as well as reduce total MAO activity, i.e. both isoforms MAO-A and MAO-B.

Increased levels of 5-HT also affect their physiology and behavior in insects of other species. For example, elevated 5-HT levels were found to significantly increase periods of sleep in *D. melanogaster* [11], and injection into the hemolymph decreased feeding in another dipteran species, the flesh fly *Neobellieria bullata* [12]. In addition, 5-HT injection into the brain of honey bees inhibited feeding, and injection into the gut excited muscle contractions, although a general elevation of 5-HT in bee hemolymph did not affect food intake [13].

Chemicals that act as neurotransmitters in the nervous system can also modulate immune function. 5-HT is such a classical neurotransmitters that also acts as an important immune regulatory molecule in both insects and mammals [14]. Qi et al. [15] report that insect hemocytes express tryptophan hydroxylase (TPH) and can synthesize 5-HT. They also note that naive hemocytes express the serotonin receptors 5-HT1B, 5-HT2B and 5-HT7. This neurotransmitter was also reported to mediate immune responses, such as hemocyte phagocytosis, nodule formation and populations of hemocyte classes in insects [16].

Insects are protected against pathogens by anatomical and physiological barriers on one level and by cellular and humoral reactions on another; however, all defensive elements are interconnected and mutually cross-regulated. For example, injury can result in the activation of humoral and cellular mechanisms and vice versa; these reactions take part in wound healing. Hemocytes can be activated by humoral factors, but they also secrete particles affecting humoral reactions [17].

These studies contribute to understanding the mechanisms underlying the interaction between innate insect immune responses and entomopathogenic metabolites. There is growing interest surrounding the use of insects as model organisms for studying the mechanisms regulating the innate immune response, which seems to be evolutionarily conserved [18].

## Results

### Effect of harman and norharman on serotonin level in *G. mellonella* larvae hemocytes

Three-day-old, last (seventh) instar *G. mellonella* larvae were given harman (H) and norharman (N) topically or mixed with food at final concentrations of 750 (1H, 1N), 1000 (2H, 2N) or 1250 (3H, 3N) ppm. Both alkaloids were also added to hemocytes cultured in vitro, and 5-HT immunolocalization was performed in all experimental groups. The level of 5-HT in whole hemolymph (containing homogenized hemocytes) was determined using ELISA. Raw data is presented in Additional file 1.

The presence of 5-HT was found in the hemocytes of the control groups, with punctate fluorescent signals observed in single cells. Serotonin concentration was found to range from 0.49 to 0.69 ng/ml of hemolymph, and hemocyte concentration increased following the administration of harman and norharman to insects.

In larvae that received the alkaloids topically, the greatest increase was found after 1 h (Fig. 1). Serotonin concentration was significantly higher (p ≤ 0.01) in all the test groups compared to controls. In the 2N, 3N, 2H and 3H groups, fluorescent signals were observed in most cells, with the highest concentrations detected in 3N (1.12 ng/ml) and 3H (1.33 ng/ml). After 24 h, elevated serotonin was found only after the topical application of norharman (Fig. 2). These levels were significantly higher than controls (p ≤ 0.01). These results were confirmed by microscopic observations.

**Fig. 1:** Serotonin in hemolymph collected from *G. mellonella* larvae 1 h after topical application of norharman and harman. **a** Immunofluorescence localization of serotonin in hemocytes. β-Actin (green) was stained by ActinGreen 488 ReadyProbes Reagent. Cell nuclei (blue) were stained with Hoechst. Serotonin (red) was detected using Mouse Serotonin Monoclonal Antibody (5HT-H209) and Goat anti-Mouse IgG (H+L) Highly Cross-Adsorbed Secondary Antibody, Alexa Fluor 594. **b** Serotonin concentration in hemolymph determined by ELISA kit. Test was performed in three independent replicates; n = 20. 1N—norharman 750 ppm, 2N—norharman 1000 ppm, 3N—norharman 1250 ppm, 1H—harman 750 ppm, 2H—harman 1000 ppm, 3H—harman 1250 ppm; ***p ≤ 0.001, **p ≤ 0.01; scale bar 25 µm

**Fig. 2:** Serotonin in hemolymph collected from *G. mellonella* larvae 24 h after topical application of norharman and harman. **a** Immunofluorescence localization of serotonin in hemocytes. β-Actin (green) was stained by ActinGreen 488 ReadyProbes Reagent. Cell nuclei (blue) were stained with Hoechst. Serotonin (red) was detected using Mouse Serotonin Monoclonal Antibody (5HT-H209) and Goat anti-Mouse IgG (H+L) Highly Cross-Adsorbed Secondary Antibody, Alexa Fluor 594. **b** Serotonin concentration in hemolymph determined by ELISA kit. Test was performed in three independent replicates; n = 20. 1N—norharman 750 ppm, 2N—norharman 1000 ppm, 3N—norharman 1250 ppm, 1H—harman 750 ppm, 2H—harman 1000 ppm, 3H—harman 1250 ppm; ***p ≤ 0.001, **p ≤ 0.01; scale bar 25 µm

Harman and norharman were also given to *G. mellonella* larvae with food. Immunolocalization and 5-HT concentration were tested in hemocytes after 24 h (Fig. 3). The most intense fluorescent signals were observed in the 2N, 3N, 1H, 2H and 3H groups, and the ELISA tests confirmed significant elevations in 5-HT level in these hemocytes compared to controls (p ≤ 0.001). The highest concentrations were detected in hemolymph after exposure to 1000 ppm harman (1.30 ng/ml) and 1250 ppm norharman (1.26 ng/ml).

**Fig. 3:** Serotonin in hemolymph collected from *G. mellonella* larvae 24 h after application norharman and harman with food. **a** Immunofluorescence localization of serotonin in hemocytes. β-Actin (green) was stained by ActinGreen 488 ReadyProbes Reagent. Cell nuclei (blue) were stained with Hoechst. Serotonin (red) was detected using Mouse Serotonin Monoclonal Antibody (5HT-H209) and Goat anti-Mouse IgG (H+L) Highly Cross-Adsorbed Secondary Antibody, Alexa Fluor 594. **b** Serotonin concentration in hemolymph determined by ELISA kit. Test was performed in three independent replicates; n = 20. 1N—norharman 750 ppm, 2N—norharman 1000 ppm, 3N—norharman 1250 ppm, 1H—harman 750 ppm, 2H—harman 1000 ppm, 3H—harman 1250 ppm; ***p ≤ 0.001; scale bar 25 µm

The effects of both alkaloids were studied also in vitro. Three concentrations of alkaloids (750, 1000 and 1250 ppm) were added to hemocyte cultures, and their effect on serotonin level was tested once after 1 h and again after 24 h. Strong fluorescence was noticed after 1 h in each tested group (Fig. 4). Serotonin was found in the majority of cells. Serotonin concentrations found to be significantly higher in the 1N, 2N, 3N, 1H, 2H and 3H groups compared to controls (p ≤ 0.001). After 24 h, no effect was observed on serotonin level in the *G. mellonella* hemocytes treated with harman (Fig. 5): although the 3H group did display slightly greater fluorescence, no significant effect on 5-HT concentration was confirmed by the ELISA test. In contrast, 5-HT concentration was increased in norharman groups 2N and 3N (p ≤ 0.01), with respective levels of 0.91 ng/ml and 0.84 ng/ml.

**Fig. 4:** Serotonin in *G. mellonella* hemocytes cultured in vitro 1 h after norharman and harman addition. **a** Immunofluorescence localization of serotonin in hemocytes. β-Actin (green) was stained by ActinGreen 488 ReadyProbes Reagent. Cell nuclei (blue) were stained with Hoechst. Serotonin (red) was detected using Mouse Serotonin Monoclonal Antibody (5HT-H209) and Goat anti-Mouse IgG (H+L) Highly Cross-Adsorbed Secondary Antibody, Alexa Fluor 594. **b** Serotonin concentration in hemolymph determined by ELISA kit. Test was performed in three independent replicates; n = 20. 1N—norharman 750 ppm, 2N—norharman 1000 ppm, 3N—norharman 1250 ppm, 1H—harman 750 ppm, 2H—harman 1000 ppm, 3H—harman 1250 ppm; ***p ≤ 0.001; scale bar 25 µm

**Fig. 5:** Serotonin in *G. mellonella* hemocytes cultured in vitro 24 h after norharman and harman addition. **a** Immunofluorescence localization of serotonin in hemocytes. β-Actin (green) was stained by ActinGreen 488 ReadyProbes Reagent. Cell nuclei (blue) were stained with Hoechst. Serotonin (red) was detected using Mouse Serotonin Monoclonal Antibody (5HT-H209) and Goat anti-Mouse IgG (H+L) Highly Cross-Adsorbed Secondary Antibody, Alexa Fluor 594. **b** Serotonin concentration in hemolymph determined by ELISA kit. Test was performed in three independent replicates; n = 20. 1N—norharman 750 ppm, 2N—norharman 1000 ppm, 3N—norharman 1250 ppm, 1H—harman 750 ppm, 2H—harman 1000 ppm, 3H—harman 1250 ppm; **p ≤ 0.01; scale bar 25 µm

### Effect of harman and norharman on phagocytosis

Phagocytic activity was examined in hemocytes obtained from *G. mellonella* larvae 1 h and 24 h after topical application and 24 h after intake with food, as well as from control insects. This process was also tested in vitro after the addition of harman or norharman directly to cell cultures. To visualize the phagocytosis process, *Escherichia coli* (K-12 strain) BioParticles fluorescein conjugate was used. Phagocytic activity was determined by measuring the resulting fluorescence, as described in “Materials and methods” section. Raw data is presented in Additional file 2.

Two types of hemocytes were visible in microscopic images: plasmatocytes and granulocytes. The remaining hemocyte subpopulations of *G. mellonella* i.e. spherulocytes, oenocytois and prohemocytes, are not adherent and were washed out during the fixation and staining procedures. Both plasmatocytes and granulocytes showed phagocytic activity. However, more intense phagocytosis was observed in granulocytes.

It was found that hemocytes from the control larvae showed phagocytic activity. In these cells, point fluorescent signals were observed. Phagocytic activity of control cells was assumed to be 100%.

An increase in phagocytic activity was observed 1 h after the topical application of harman and norharman (Fig. 6). Significantly stronger fluorescence intensity was found in the 1N, 2N, 3N, 1H, 2H, 3H groups compared to controls. These observations confirmed the quantitative data. A statistically significant (p ≤ 0.001) increase in the amount of phagocytized *E. coli* bioparticles was detected. The highest relative phagocytosis values were measured in the 3N (182.6%) and 3H (183.3%) groups. No effect was observed 24 h after topical application (Fig. 7). Slightly greater fluorescence was observed in the 1N, 2N and 3N groups; however, no statistically significant differences in phagocytic activity were found compared to controls.

**Fig. 6:** Phagocytic activity of *G. mellonella* hemocytes 1 h after topical application of norharman and harman. **a** Immunofluorescence localization of phagocytized *E. coli* bioparticles in hemocytes. β-Actin (orange) was stained by ActinRed™ 555 ReadyProbes Reagent. Cell nuclei (blue) were stained with Hoechst. To visualize the phagocytosis of hemocytes the *Escherichia coli* (K-12 strain) BioParticles fluorescein (green) conjugate (Invitrogen) were used. **b** Relative phagocytosis. The data are expressed as the percentage of phagocytosis compared with control values (100%). Test was performed in three independent replicates; n = 20. 1N—norharman 750 ppm, 2N—norharman 1000 ppm, 3N—norharman 1250 ppm, 1H—harman 750 ppm, 2H—harman 1000 ppm, 3H—harman 1250 ppm; ***p ≤ 0.001; scale bar 25 µm

**Fig. 7:** Phagocytic activity of *G. mellonella* hemocytes 24 h after topical application of norharman and harman. **a** Immunofluorescence localization of phagocytized *E. coli* bioparticles in hemocytes. β—actin (orange) was stained by ActinRed™ 555 ReadyProbes Reagent. Cell nuclei (blue) were stained with Hoechst. To visualize the phagocytosis of hemocytes the *Escherichia coli* (K-12 strain) BioParticles fluorescein (green) conjugate (Invitrogen) were used. **b** Relative phagocytosis. The data are expressed as the percentage of phagocytosis compared with control values (100%). Test was performed in three independent replicates; n = 20. 1N—norharman 750 ppm, 2N—norharman 1000 ppm, 3N—norharman 1250 ppm, 1H—harman 750 ppm, 2H—harman 1000 ppm, 3H—harman 1250 ppm; scale bar 25 µm

A significant change in hemocyte phagocytic activity was observed in the larvae administered harman and norharman with food (Fig. 8). After 24 h, a significant increase in fluorescence intensity was observed in all analyzed groups (p ≤ 0.05).

**Fig. 8:** Phagocytic activity of *G. mellonella* hemocytes 24 h after application of norharman and harman with food. **a** Immunofluorescence localization of phagocytized *E. coli* bioparticles in hemocytes. β-Actin (orange) was stained by ActinRed™ 555 ReadyProbes Reagent. Cell nuclei (blue) were stained with Hoechst. To visualize the phagocytosis of hemocytes the *Escherichia coli* (K-12 strain) BioParticles fluorescein (green) conjugate (Invitrogen) were used. **b** Relative phagocytosis. The data are expressed as the percentage of phagocytosis compared with control values (100%). Test was performed in three independent replicates; n = 20. 1N—norharman 750 ppm, 2N—norharman 1000 ppm, 3N—norharman 1250 ppm, 1H—harman 750 ppm, 2H—harman 1000 ppm, 3H—harman 1250 ppm; *p ≤ 0.05; **p ≤ 0.01; ***p ≤ 0.001; scale bar 25 µm

The effects of these alkaloids was also examined in vitro. One hour after addition, strong fluorescence signals were reported for all examined groups (Fig. 9). The quantitative measurements showed that fluorescence was significantly higher (p ≤ 0.001) than in the controls. The highest values of relative phagocytosis were found in 3H (174.1%) and 3N (187.7%) samples. After 24 h, the alkaloids displayed a more diversified effect on phagocytosis (Fig. 10), with norharman having a stronger effect on in vitro phagocytic activity, and more intense fluorescence being observed in the 1N, 2N and 3N groups compared to controls. This was correlated with a significantly (p ≤ 0.001) higher measurement of relative phagocytosis. Harman only induced a significant increase in phagocytic activity when given at a concentration of 1000 ppm (group 2H) (p ≤ 0.05).

**Fig. 9:** Phagocytic activity of *G. mellonella* hemocytes in vitro 1 h after norharman and harman treatment. **a** Immunofluorescence localization of phagocytized *E. coli* bioparticles in hemocytes. β-Actin (orange) was stained by ActinRed™ 555 ReadyProbes Reagent. Cell nuclei (blue) were stained with Hoechst. To visualize the phagocytosis of hemocytes the *Escherichia coli* (K-12 strain) BioParticles fluorescein (green) conjugate (Invitrogen) were used. **b** Relative phagocytosis. The data are expressed as the percentage of phagocytosis compared with control values (100%). Test was performed in three independent replicates; n = 20. 1N—norharman 750 ppm, 2N—norharman 1000 ppm, 3N—norharman 1250 ppm, 1H—harman 750 ppm, 2H—harman 1000 ppm, 3H—harman 1250 ppm; ***p ≤ 0.001; scale bar 25 µm

**Fig. 10:** Phagocytic activity of *G. mellonella* hemocytes in vitro 24 h after norharman and harman treatment. **a** Immunofluorescence localization of phagocytized *E. coli* bioparticles in hemocytes. β-Actin (orange) was stained by ActinRed™ 555 ReadyProbes Reagent. Cell nuclei (blue) were stained with Hoechst. To visualize the phagocytosis of hemocytes the *Escherichia coli* (K-12 strain) BioParticles fluorescein (green) conjugate (Invitrogen) were used. **b** Relative phagocytosis. The data are expressed as the percentage of phagocytosis compared with control values (100%). Test was performed in three independent replicates; n = 20. 1N—norharman 750 ppm, 2N—norharman 1000 ppm, 3N—norharman 1250 ppm, 1H—harman 750 ppm, 2H—harman 1000 ppm, 3H—harman 1250 ppm; *p ≤ 0.05; **p ≤ 0.01; ***p ≤ 0.001; scale bar 25 µm

### The influence of harman and norharman on cytoskeleton organization in hemocytes

The effect on harman and norharman on hemocyte cell morphology was documented after 24-h in vitro cultivation. As only plasmatocytes and granulocytes were strongly attached to the slide surface and were not washed out during the fluorescence dyeing, only these were visible in the microscope images.

The cellular networks were visible in the images of the control groups (Figs. 1, 2, 3, 4, 5, 6, 7, 8, 9, 10).

During the course of in vitro hemocyte culture, the plasmatocytes become elongated, formed numerous pseudopodial and filopodial structures, actively moved towards the neighboring plasmatocytes and formed networks with them. Granulocytes were included in the networks formed by plasmatocytes.

Harman and norharman had an impact on cytoskeleton organization. Changes in cell structure were observed after 1250 ppm alkaloid treatment, both topically and with food (Figs. 1, 2, 3 and 6, 7, 8). Inhibition of network formation by plasamatocytes and granulocytes was also observed in the in vitro hemocyte cultures treated with 1000 and 1250 ppm alkaloid (Figs. 4, 5, 9, 10). More detailed changes in hemocyte structure such as abnormal form, naked nuclei, cell aggregates, fragments of disintegrated cells, interrupted cell membrane continuity and actin condensation in cells are given in Fig. 11.

**Fig. 11:** Changes in cytoskeleton organization in hemocytes from *G. mellonella* larvae treated with harman or norharman. β-Actin (red) was stained by ActinRed 488 ReadyProbes Reagent. Cell nuclei (blue) were stained with Hoechst. **a** Abnormal cell shape, **b** naked nuclei (marked with an arrows), **c** cell aggregates, **d** fragments of disintegrated cells, **e** interrupted cell membrane continuity, **f** actin condensation. Scale bar 10 µm

## Discussion

Although the β-carboline alkaloids harman and norharman are known to have metabolic properties in plants, their effect on mammalian organisms is less understood. Both substances are reversible competitive monoamine oxidase (MAO) inhibitors, with norharman preferentially inhibiting MAO-B and harman inhibiting MAO-A; the two are considered to be the strongest inhibitors of MAO [19]. MAO is an intramitochondrial enzyme responsible for the breakdown of intracellular dopamine, norepinephrine and serotonin, and its inhibition results in an increase in monoamine concentration [20].

Harman and norharman are also known to serve as fungal metabolites, and have previously been found to be secreted by the entomopathogenic fungus *C. coronatus* propagated in liquid minimal medium (MM) and rich medium (LB). Higher concentration was detected in LB medium. The insect’s body is a very rich source of nutrients for parasitic fungi, much richer than the LB medium. After infection of the insect host by *C. coronatus*, the fungus can produce a range of compounds in the insect, including these alkaloids, at concentrations which may significantly differ from those observed in the in vitro cultures.

Harman and norharman administration increased the serotonin concentration in the heads of *G. mellonella* larvae, an important pest of beehives, and significantly decreased MAO-A concentration and total MAO activity in larval tissues 1 h after administration. As in the present work, harman and norharman were administered topically and with food in three concentrations: 750, 1000 and 1250 ppm [10].

Following on from these findings, the current work examines whether these alkaloids may also affect serotonin concentration in *G. mellonella* hemocytes and their phagocytic activity.

Our findings indicate that 24 h of exposure to food contaminated with harman and norharman resulted in significant increases in serotonin level and hemocyte phagocytic activity. Similar responses were noticed 1 h after topical application or addition to in vitro hemocyte culture; however, these responses were found to decrease 24 h later, suggesting decomposition or exertion of alkaloids or serotonin. The mechanisms of harman and norharman metabolism in insects are presently unknown.

Herr et al. [21] report that human macrophages can degrade 5-HT. In insects, the metabolism of serotonin is partially recognized in the nervous system but completely unknown in the immune system. The primary catabolic pathway for biogenic amines is oxidative deamination by monoamine oxidase (MAO). Enzymatic inactivation in invertebrates is thought to take place after amino-terminal tagging with specific groups, mainly *N*-acetylation or *N*-methylation; however, γ-glutamylation, sulphation, and β-alanyl conjugation are also possible [22].

From an evolutionary perspective, serotonin is one of the oldest substances found in animals [23]. This neurotransmitter regulates many processes in both vertebrates and invertebrates: locomotion, reproduction, learning and memory, behavior including pain, appetite, mood and sleep [24]. In addition to its widely-understood effects on the nervous system, 5-HT also acts on the immune system; however, this effect is recognized mainly in mammals. Immune cells express the serotonin receptors 5-HT1, 5-HT2, 5-HT3, 5-HT4 and 5-HT7 and the serotonin transporter (SERT), as well as the key enzymes for serotonin synthesis (tryptophan hydroxylase-TPH) and for serotonin degradation (MAO) [21]. Serotonin is also known to exert functions in innate as well as adaptive immunity: Sternberg et al. [25, 26] found serotonin to have inhibitory or stimulatory effects on murine macrophages, depending on the dose. Serotonin suppressed interferon (IFN-)γ-induced phagocytosis and the expression of class II MHC [26]. 5-HT was found to block interactions between monocytes and NK cells, leading to an increase of NK cell functions that are typically inhibited by monocytes, such as cytotoxicity and IFN-γ production [27], and serotonin depletion has been associated with reduced splenic T cell proliferation in following concanavalin A treatment [28]. In addition, 5-HT may also modulate cytokine secretion. Dürk et al. [29] note that serotonin modulated the release of cytokines IL-1β, IL-6, IL-8/CXCL8, IL-12p40 and TNF-α in LPS-stimulated human blood monocytes, while Müller et al. [30] report that serotonin induces oriented migration of immature dendritic cells and upregulates the production of IL-6.

A decrease in the production of reactive oxygen species (ROS) has also been observed in neutrophils following serotonergic stimulation [31–33]. In addition, serotonin induces eosinophil trafficking and recruitment [34], and local secretion of serotonin from platelets has been found to initiate T cell-dependent interaction sensitivity mediated by IgE antibodies [35]. Mitogen-stimulated B-cell proliferation has also been found to be dependent on serotonin stimulation via the 5-HT1A receptor [36].

Insect immune systems show a high degree of structural and functional homology to the innate immune systems of mammals. Even so, the insect immune response generally differs from vertebrates in that it lacks immunoglobulins and memory; however, insects demonstrate an innate non-adaptive defense reaction that exhibits striking similarities to the vertebrate acute-phase response [18]. The innate immune system of insects contains physical barriers, such as the exoskeleton, trachea structure and peritrophic membrane, which are supported by humoral responses and cellular responses. The humoral response consists of soluble effector molecules such as opsonins, melanin, prophenoloxidase cascade, and antimicrobial peptides (AMPs), while cellular immunity comprises hemocyte-mediated reactions such as phagocytosis, nodule formation, encapsulation and clotting [37, 38]. Both types of immune response, humoral and cellular, participate in wound healing in reaction to injury and in the neutralization of pathogens.

*Galleria mellonella* larvae are often used as a model in the study of the immune system. There are five classes of hemocytes in the hemolymph of these insects, the largest being adherent granulocytes and plasmatocytes, with the remainder comprising non-adhesive spherule cells, prohemocytes and oenocytoids. Plasmatocytes form capsules around foreign bodies which are too large to be phagocytosed, or nodules around many types of bacteria and necrotic melanised material. During these processes, plasmatocytes synthesize numerous desmosomes and contain large amounts of microtubules in their cytoplasm [39]. The role of plasmatocytes in phagocytosis in Lepidoptera is unclear. Our studies have shown that plasmatocytes have phagocytic activity in *G. mellonella*, however, this process was not intensive, with only some cells being phagocytosed. Some authors regard both plasmatocytes and granulocytes as phagocytes [40–42], while others indicate that plasmatocytes are evidently not phagocytic cells [43–45]. In addition, some literature data suggests that only plasmatocytes are active phagocytes [46, 47]. These differences may result from variations in the cell culture conditions, as hemocyte function may depend on the composition of medium, the method of hemolymph collection and incubation time. Boguś et al. [48] indicate the presence of only one type of plasmatocyte in fresh hemolymph in *G. mellonella*, but of three types after 24-h incubation.

One of the main functions of granulocytes is phagocytosis. Granular hemocytes have also been shown to be the first cells to come into contact with a pathogen at the beginning of capsule/nodule formation. After contact with the foreign body, they eject their granular content [49]. This exocytosis of typical inclusions by granulocytes supports the influx of plasmatocytes or at least helps plasmatocytes construct the capsule or nodule [50]. Our present findings confirm that granulocytes from *G. mellonella* larvae are phagocytic cells, and that this process was stronger than in plasmatocytes.

The main function of oenocytoids is the synthesis of phenoloxidase (PO): the substance responsible hemolymph darkening by melanin synthesis [51]. The functions of spherule cells are totally unknown in Lepidoptera [52].

Harman and norharman were found to influence the cytoskeletons of *G. mellonella* plasmatocytes and granulocytes, with disturbances in hemocyte network formation being observed, as well as abnormal cell shape, naked nuclei, cells aggregates, fragments of disintegrated cells, interrupted cell membrane continuity and actin condensation in cells. Although no studies have so far examined the effect of β-carboline alkaloids on the morphology of insect hemocytes, it is known that the wax moth hemocyte cytoskeleton is influenced by infection with *C. coronatus*, whose metabolites are harman and norharman. Widespread cell vacuolization and large numbers of disintegrated granulocytes were observed in the hemolymph after 24-h incubation with fungus, while all hemocytes were found to be fragmented in the dying insects 48 h after exposure [48].

A common feature of the immune cells of mammals and insects is the occurrence of serotonin receptors. Qi et al. [15] identified 5-HT1B, 5-HT2B, and 5-HT7 receptor expression in naive insect hemocytes, but only 5-HT1B and 5-HT2B appeared to have functional roles. While blockade of 5-HT1B significantly reduced phagocytic ability, blockade of 5-HT2B increased hemocyte phagocytosis. Harman and norharman are antagonists of both type 5-HT1 and 5-HT2 serotonin receptors, and both increase serotonin levels by acting as MAO inhibitors. This may explain our present findings, which show that harman and norharman administration results in an increase of 5-HT in the hemolymph and elevated phagocytic activity by hemocytes. Other authors have also found that serotonin can modulate phagocytosis in insects. Baines et al. [53] report that octopamine and 5-hydroxytryptamine (5-HT) increase phagocytosis in vitro in cockroach (*Periplaneta americana*) hemocytes, while Kim et al. [54] note that octopamine or 5-HT markedly enhanced both hemocytic phagocytosis and nodule formation in *Spodoptera exigua* larvae.

As *C. coronatus* has been found to express harman and norharman as [10], our research suggests that entomopathogenic fungi can modulate the immune response of insects. Kędra and Boguś [49] report that *C. coronatus* infection increased the phagocytic activity of *G. mellonella* plasmatocytes by 3.3 times and of *Dendrolimus pini* plasmatocytes by 2.1 times. In contrast, plasmatocytes of *G. mellonella* larvae were found to display pathogenic changes in cytoskeleton structure and decreased phagocytic activity following infection with *Metarhizium anisopliae* or *Bauveria bassiana* fungi [55, 56].

As fungal spores and fragments of hyphae are too large to be phagocytized [57], the two main cellular immunological processes employed by insects to limit fungal infection are nodulation and encapsulation. It is possible, then, that some entomopathogenic fungi may win an advantage by redirecting the potency of the insect immune system away from nodulation and encapsulation, and toward the phagocytosis process. However, further studies are required to confirm, or refute, this hypothesis.

## Conclusion

The results of this innovative study may have a considerable impact on research concerning insect physiology, parasitology, immunology and biocontrol of pests. Our initial findings confirm that harman and norharman, expressed as metabolites of the entomopathogenic fungus *C. coronatus* may stimulate the phagocytic activity of *G. mellonella* hemocytes by elevating serotonin levels; however, further research is needed to obtain a deeper insight into the molecular basis of this poorly-understood phenomenon.

## Materials and methods

### Insects

A culture of the wax moth, *G. mellonella* (Lepidoptera) was maintained and reared in constant darkness on an artificial diet [58] in chambers with controlled temperature and humidity (30 °C, 70% r.h). Three-day-old last instar larvae were used for analyzing the influence of harman and norharman on insects and their defense system.

### Harman and norharman application

Harman and norharman (Sigma-Aldrich) were administered to the *G. mellonella* larvae by topical application and in the diet at final concentrations based on Wrońska et al. [10] The alkaloids were diluted in acetone for topical applications, where each larva received 5 µl of harman or norharman solution containing 750, 1000 or 1250 ppm of the appropriate alkaloid.

For intake with food, harman and norharman were dissolved in 5% methanol in distilled water, and 5 ml of each alkaloid solution was incorporated into 5 g of insect food to achieve a final concentration of 750, 1000 or 1250 ppm, respectively. The solvent was then evaporated from the food at 35 °C in an oven for 48 h. Before the addition of alkaloid, the food itself was baked at 180 °C for 1 h to dry it and to kill any bacteria which might be pathogenic for the insects. The food was prepared once for whole experiment.

The larvae consumed the treated food throughout the entire experiment. The control group consisted of insects fed with food treated with solvent instead of alkaloids. All harman and norharman application, both topical and dietary was performed in 3-day-old final (seventh) instar larvae. At this stage, the larvae were not only large enough for precise sample collection but were also still feeding: the cessation of physiological feeding prior to metamorphosis takes place on the fifth to sixth day of the final instar [59].

### Larval hemolymph collection and hemocyte culture

*Galleria mellonella* hemolymph was collected from both control larvae and those treated with alkaloid: either 1 h and 24 h after topical application or 24 h after intake with food). No samples were taken 1 h after dietary administration of alkaloids as this period was too short to be sure that all larvae had started eating food contaminated with alkaloids: *G. mellonella* larvae consume food with varying intensity. Before bleeding, larvae were washed with distilled water and then immersed briefly in 70% (v/v) ethanol to sterilize their surfaces, thus reducing the contamination of hemolymph samples. Hemolymph was taken from the larvae through an incision made in the last proleg. Freely-dripping hemolymph was collected into sterile polypropylene 1.5 ml centrifuge tubes preloaded with 300 µl of Grace’s Insect Medium (GIM; Gibco) with added gentamycin (10 mg/ml; Gibco), amphotericin B (250 µg/ml; Gibco) and phenylothiourea (PTU; 0,1 mM; Sigma-Aldrich). The hemolymph suspensions were immediately used for cell culture or frozen at − 80 °C.

For hemocyte culture, hemolymph mix (100 μl of fresh hemolymph collected from ten larvae in 500 μl of supplemented GIM) was transferred to a six-channel μ-Slide IV 0.4 (IBIDI)—100 μl for each channel. The slides were incubated in 30 °C for 24 h.

To study the effect of harman and norharman on hemocytes in vitro, alkaloids were added to cell culture at final concentrations of 750 ppm, 1000 ppm and 1250 ppm. The cells were cultured with the alkaloids for 1 h and 24 h in 30 °C. Each culture was performed in three independent replicates, with ten larvae used for each instance.

### Serotonin (5-HT) detection

Immunolocalization of serotonin (5-HT) was performed in all hemocyte cultures. The cells were fixed in 4% Paraformaldehyde (Sigma-Aldrich; PFA) in Phosphate-buffered saline (PBS) and permeabilized in 0.1% Triton X-100 (Sigma-Aldrich) in PBS. The cells were incubated overnight at 4 °C with Mouse Serotonin Monoclonal Antibody (5HT-H209) (Invitrogen), the primary antibody, which was diluted 1:40 in PBS with 1% bovine serum albumin (BSA). The cells were then incubated in 4% BSA-PBS for 2 h to prevent non-specific antibody binding. Following this, the hemocytes were incubated for a further 2 h at room temperature with secondary antibody Goat anti-Mouse IgG (H+L) Highly Cross-Adsorbed Secondary Antibody, Alexa Fluor 594 (Invitrogen) in concentration 2 µg/ml. ActinGreen™ 555 ReadyProbes Reagent (Invitrogen) was used to label the actin fibers. The cell nuclei were stained with Hoechst (Enzo Life Sciences). The hemocytes were observed under an Axio Vert.A1 fluorescence microscope (Zeiss) with Axio Cam ICc 5 (Zeiss) and ZEN lite 2012 software.

The amount of 5-HT in *G. mellonella* larval hemolymph was also determined. Hemolymph from the treated larvae was collected as described above.

The concentration of serotonin was investigated also in hemocyte cultures in vitro. After incubation with alkaloids, cells were detached by trypsin–EDTA solution 0.25% (Gibco), and the cell suspensions were transferred to sterile polypropylene 1.5 ml centrifuge tubes. The samples were homogenized by sonication and centrifuged at 250×*g* for 10 min at 4 °C. The supernatants were stored at − 80 °C. The level of 5-HT present in the supernatants was determined using a commercial ELISA kit produced by Labor Diagnostika Nord (LDN), (Germany). Each test was performed in three independent replicates.

### Phagocytic activity

Phagocytic activity was examined in hemocytes collected from *G. mellonella* larvae 1 h and 24 h after topical application, 24 h after intake with food, as well as from control insects. This process was also tested in vitro following the direct addition of harman or norharman to cell cultures. Each test was performed in three independent replicates.

The phagocytic activity of the hemocytes was visualized by examining their action against *Escherichia coli* (K-12 strain) BioParticles using fluorescein conjugate (Invitrogen). The cells were cultured as described above. After 24-h incubation with the *E. coli* bioparticles, the cells were fixed in 4% PFA–PBS (phosphate-buffered saline PBS, paraformaldehyde PFA) and permeabilized in 0.1% Triton X-100 in PBS. ActinRed™ 555 ReadyProbes Reagent (Invitrogen) was used to label the actin fibers. The cell nuclei were stained with Hoechst (Enzo). The obtained samples were analyzed by Axio Vert.A1 fluorescence microscope (Zeiss) with Axio Cam ICc 5 (Zeiss) and ZEN lite 2012 software.

Phagocytic activity was also quantified. After 24-h incubation with *E. coli* bioparticles, the cells were fixed in 4% PFA–PBS, and their fluorescence (Ex = 494 nm, Em = 518 nm) was measured using a Synergy HT Multi-Detection Microplate Reader (BioTek). The level of fluorescence was proportional to the amount of phagocytized particles. The results are expressed as the percentage of phagocytosis compared with control values (100%).

### Statistics

The normality of the data was tested using the Kolmogorov–Smirnov test. The t-test for independent samples was used to compare the results of the control group and the study group. The results were regarded as being statistically significant at p ≤ 0.05. STATISTICA 6.1 software (StatSoft Polska) was used for all calculations.

## Additional files

**Additional file 1: Table S1.** Serotonin concentration [ng/ml] in hemolymph collected from *G. mellonella* larvae after application of norharman and harman-raw data. 1N—norharman 750 ppm, 2N—norharman 1000 ppm, 3N—norharman 1250 ppm, 1H—harman 750 ppm, 2H—harman 1000 ppm, 3H—harman 1250 ppm.

**Additional file 2: Table S2.** Phagocytic activity of *G. mellonella* hemocytes after application of norharman and harman—raw data. The data are expressed as the percentage of phagocytosis compared with control values (100%). 1N—norharman 750 ppm, 2N—norharman 1000 ppm, 3N—norharman 1250 ppm, 1H—harman 750 ppm, 2H—harman 1000 ppm, 3H—harman 1250 ppm.
